The article "Dose institutional quality influences the relationship between urbanization and CO2 emissions?" was retracted in 2025. Reasons: concerns about the results or conclusions; concerns about the peer review; concerns about the authorship.

# Dose institutional quality influences the relationship between urbanization and CO2 emissions?

**DOI:** 10.1371/journal.pone.0291930

**Published:** 2023-10-11

**Authors:** Hayat Khan, Tengpeng Chen, Robeena Bibi, Itbar Khan

**Affiliations:** 1 School of Economics and Management, Zhejiang University of Science and Technology, Hangzhou, China; 2 China Center for Special Economic Zone Research, Shenzhen University, Shenzhen, China; 3 School of Public Administration, Hohai University, Nanjing, China; 4 College of Economics, Shenzhen University, Shenzhen, China; National University of Sciences and Technology, PAKISTAN

## Abstract

As a result of rapid economic expansion, increased energy use, and urbanization, global warming and climate change have become serious challenges in recent decades. Institutional quality can be the remedy to impede the harmful effect of factors on environmental quality. This study investigates the impact that urbanization and institutional quality on environmental quality in in the Belt and Road Initiative (BRI) countries from 2002 to 2019. By using two step generalized method of moment, the findings shows that urbanization leads to an increase in carbon dioxide emissions and a decline in environmental quality. On the other hand, the square term of urbanization indicates that an increase in urbanization leads to a reduction in emissions at a later stage after reach a certain level. Education, on the other hand, has the reverse impact of increasing carbon emissions; economic growth, foreign direct investment, and government effectiveness all boost carbon emissions. In a similar vein, the interaction between urbanization and the effectiveness of the government is unfavorable, underscoring the transformative role that the effectiveness of the government plays in leading to environmental sustainability. Finally, the findings of this study have considerable policy implication for the sample countries.

## Introduction

Several factors, such as economic globalization, economic growth, and energy consumption, are associated with carbon dioxide emissions, and an increase in these factors influences the quality of the environment. Same like other factors, urbanization also affects environmental quality, where some studies in the prevailing literature indicate that a rise in long term economic growth improves environmental quality. However, a rise in urban populations increases environmental degradation Adem, Solomon [1]. Cities in a country are widely regarded as the primary sources of carbon emissions due to increased urbanization. Economic growth is important for a country, specifically for developing and emerging countries. These countries are increasing economic activities to raise growth and living standards as required by developing countries, but this leads to lower environmental quality by increasing carbon dioxide emissions. The economic activities may require high industrialization, production, and the use of energy from fossil fuels, which are harmful to the quality of environment. Urbanization also facilitates economic development as it creates forces of market demand that accompany the use of energy and carbon dioxide emissions. The adaptation of industrial structures in urban development, as well as the rise in urbanization, increase the use of energy, resulting in high carbon emission discharge Glaeser and Kahn [2]. An another study confirms this statement that the level of urbanization raise carbon dioxide emissions and worsen the quality of the environment Sadorsky [3]. On the other hand, contrary findings are obtained shows that low population density causes inefficient public transportation and infrastructure, reducing carbon emissions Chen, Colombo [4]. Similarly, Muñoz, Zwick [5] identified the lowest carbon footprint in urban areas, while Zhang, Wang [6] stated that urbanization in an economy has been considered concerning scale effect and the driving factor of development with the use of environmental friendly energy. Most of these developing and emerging countries focus on raising economic growth, which raises carbon dioxide emission and worsens environmental quality. Foreign direct investment is also associated with environmental quality in two aspects, the pollution halo, and the pollution haven effect. The halo hypothesis indicates that foreign direct investment reduces emissions and raises environmental quality, while the Haven effect has the opposite effect. These effects depend on the level of foreign direct investment policies and institutions in a country. The harmful effect of these economic factors and the level of urbanization on carbon dioxide can be linked to the quality of institutions in a country, especially the government’s effectiveness. The level of education in a country can also play an important role in enhancing environmental quality. Consequently, it’s important to examine the effect of education and government effectiveness in the linkage of urbanization and carbon dioxide emission.

The article "Dose institutional quality influences the relationship between urbanization and CO2 emissions?" was retracted in 2025. Reasons: concerns about the results or conclusions; concerns about the peer review; concerns about the authorship.

The nexus between urbanization and carbon dioxide has been established and analyzed in previous studies, although no consistent conclusion has been reached. The role of government effectiveness and education has not been included, while only the direct effect of urbanization has been studied; the nonlinear association between urbanization and carbon dioxide has not been explored, which needs attention. Likewise, this study included the interaction term between government effectiveness and urbanization, which is new and unique in such a study. The relationship between urbanization and carbon emissions can be examined using the transformative role of government effectiveness. Some studies have been conducted on developing countries and developed countries, and so on; however, considering the unique characteristics of the belt and road countries such as urbanization level, economy, trade, and institutions, no studies have been done on this association. The current study examines the nexus between urbanization and carbon dioxide. The belt and road countries must address governance, social, and economic challenges together. Most of the Belt and Road countries are emerging and developing countries, and this study analyzed the objectives in this sample countries, which are highly suitable and representative in this context as these countries are still focusing on rising economic growth and there is an increasing urbanization. The main objective of this study is to examine the nexus between urbanization and carbon emissions by introducing government effectiveness into this relationship. Important policies can be suggested to the sample countries by investigating this association about urbanization, government effectiveness, and environmental quality. Considering the above points, this study explores both the direct and nonlinear nexus of urbanization with carbon dioxide by taking into consideration the moderating role of government effectiveness in this association. Data for 39 belt and road countries have been taken for the years 2002–2020 based on the availability of data and employing dynamic panel models for analysis. The stationarity of data was first checked by the second-generation panel unit root tests, and then static and dynamic models were applied for analysis. According to the findings, urbanization increases carbon dioxide emissions, and there is a U-shaped relationship between urbanization and emissions. Foreign direct investment and economic growth also increase carbon dioxide, while education reduces environmental degradation. On the other hand, the interactive term between urbanization and institutions confirms that there is a moderating role for government effectiveness in the nexus between urbanization and carbon dioxide.

The remaining parts of the study is structured in this sequence. Part 2 is composed of a literature review, Part 3 is composed of methods and variables used, Part 4 presents results, and Part 5 gives recommendations and a conclusion.

## Literature review

### Urbanization and carbon dioxide emission

Several investigations on the link between urbanization and carbon dioxide emissions have been given in the prior research, and these studies have arrived at a variety of conclusions depending on the country in which they were conducted. It is generally accepted that urbanization is a process in which the majority of the working population shifts from being farmers to residents of non-rural areas, leading to an increase in the number of people living in cities. Urbanization is quickly becoming the most major socioeconomic shift taking place anywhere in the world, particularly in countries that are still developing [7]. The inevitable result of social progress, economic growth, and technological improvement is urbanization. This trend cannot be stopped. The level of urbanization in a country or region is a good indicator of the country’s or territory’s socioeconomic development. As a result of the fact that a city frequently acts as an economic center, it is responsible for the economic growth of neighboring regions, and the improvement in the degree of economic development in the region in turn encourages the expansion of the city. The urbanization of China has been a significant development on a worldwide scale. [8] demonstrate that urbanization does not affect environmental quality when rigorous environmental standards are in place. [9] utilized data for thirty different Chinese provinces spanning the years 2000 to 2016. The authors found that there is a link that looks like the letter U between urbanization and carbon dioxide emissions. The information used in this study was gathered between the years 2000 and 2016. Research with the same design but carried out on a variety of samples produced contrasting findings. According to [10] for example, fast urbanization causes a rise in carbon dioxide emissions and a decline in the quality of the ecosystem. Urbanization is associated with an increase in economic activity, which in turn is associated with an increase in carbon dioxide emissions. Research of a similar nature was carried out [11] who investigated the effect that urbanization has on carbon dioxide emissions by analyzing data spanning the years 1975 to 2015 for a number of country groupings. The authors came to the conclusion that different income groups experience varying degrees of impact from urbanization throughout time. [12] studied urbanization in China. The data point to a relationship that is formed like a U between urbanization and the degradation of the natural environment. [13] studied the nexus between urbanization, energy demand and road infrastructure in Pakistan from 1971 to 2018 using VECM model. The findings show a positive contribution of urbanization to energy consumption in road sector. [14] studied the impact of economic growth and urbanization on environmental quality in western Africa from 1981 to 2018 using Driscoll-Kraay panel regression. The findings shows that manufacturing value added, urbanization, FDI and financial development increase environmental degradation. [15] studied the nexus between natural resources abundance, urbanization and environmental degradation in China. The authors employed Bayer and Hack cointegration test, and bootstrap causality technique to study cointegration where the findings shows that there exists long run equilibrium among variables. The findings illustrate that natural resources rent rise ecological footprint where urbanization and economic growth contribute to environmental degradation. Ahmed explores the non-linear association between urbanization and carbon emission from 1971 to 2014 in Indonesia. The findings shows that there is an inverted shaped association between urbanization and carbon emission. An increase in urbanization raises carbon dioxide emission but its reduce emission after a certain level. Economic growth and energy intensity also rise emission while there is no effect of trad openness on carbon emission.

The article "Dose institutional quality influences the relationship between urbanization and CO2 emissions?" was retracted in 2025. Reasons: concerns about the results or conclusions; concerns about the peer review; concerns about the authorship.

### Institutional quality, urbanization, and carbon dioxide emission

This association can be linked to the role that institutions play, such as the part that the government plays. Perceptions of the quality of public services, the quality of the civil service and the degree to which it is independent from political pressures, the quality of policy formulation and implementation, and the credibility of a government’s commitment to such policies are all components that make up the definition of government effectiveness [16]. Because of the rapid expansion of the contemporary economy, urbanization can also have an impact on the efficiency of government, which in turn plays a significant role in the production of carbon emissions. On the one hand, urbanization fosters system stability, the advancement of technology, and the enhancement of the quality of the population, all of which are the foundation for improving the efficiency of the government. On the other hand, urbanization has the opposite effect and reduces the quality of the population. To be more specific, the application of technology in the development of smart cities has the potential to considerably boost the effectiveness of governance. On the other hand, the development of urbanization, the migration of population from rural to urban areas, economic and social construction, and the emergence of innovations will place greater demands on the governance level of the economic system, social mechanisms, relevant laws, and regulations, and urban construction, which will necessitate the improvement of a government’s efficacy. This is because urbanization, the migration of population from rural to urban areas, economic and social construction, and the emergence of innovations will place greater demands on the governance level of People have been able to steadily meet their fundamental needs and improve their living conditions as a result of urbanization. As a result, they are now seeking a greater degree of satisfaction regarding their welfare, which necessitates an increase in the quality of the services provided by the government. There haven’t been many research that look at the connections between urbanization and the effectiveness of governance. Using QARDL and data ranging from 1995 to 2018, [17] investigated the relationship that exists between institutions, information and communication technologies, and carbon emissions. According to the findings of the study, economic expansion and the presence of institutions both contribute to a rise in carbon dioxide emissions, although the use of information and communications technology works to reduce emissions. Using OLS, fixed effects, and the generalized method of moments estimators [18] investigated the role of institutional quality and financial development in environmental sustainability in the belt and road countries from 1985 to 2019. This research covered the time period from 1985 to 2019. According to the findings, three out of the six variables of institutional quality, namely the efficacy of government, voice and accountability, and control of corruption, all contribute to a rise in carbon dioxide emissions. On the other hand, quality regulation, the rule of law, and political stability all contribute greatly to a reduction in carbon dioxide emissions and an improvement in environmental quality. The researchers [19] investigate the influence that institutional quality plays in lowering carbon emissions in BRI, developing, and global panel nations between the years 2002 and 2019. The authors found that institutional quality positively affected FDI inflow using OLS, fixed effect, and dynamic GMM models. On the other hand, governance indicators were poor in all panels, such as regulatory quality, rule of law, and political stability; accountability and control of corruption were weak indicators to reduce emissions in BRI countries. [20] conducted research to investigate the relationship between Chile’s economic growth, carbon emissions, the quality of the country’s institutions, and foreign direct investment. Both the positive and negative effects of economic growth, institutional quality, and renewable energy have both positive and negative effects on the environment. These effects have favorable benefits on the environment since they decrease emissions, whereas the negative effects increase emissions. In contrast, both the positive and negative effects of foreign direct investment and fossil fuels would have a negative influence on the environment of Chile by raising carbon emissions. This would be due to the fact that both of these factors would increase the demand for fossil fuels. [21] conducted research in Asian nations to determine the connection between foreign direct investment (FDI), institutional quality, and carbon emissions. As an example, they used Japan. They came to the conclusion that the consumption of energy has a detrimental effect on greenhouse gas emissions, and that the quality of regulation in Asia contributes to a rise in greenhouse gas emissions. They also found information regarding investments made by foreign governments in order to improve energy conservation and the use of sustainable energy. On the other hand, [22] evaluated the effect that institutional quality and the use of renewable energy had on carbon emissions in developing nations between the years 1995 and 2017. Models of the MG, AMG, CCEMG, and GMM families were used. They made the discovery that the standard of the institutions can put a cap on the amount of energy used and increase the efficiency with which it reduces carbon emissions. Both the quality of their institutions and the amount of energy they use have a detrimental and considerable impact on the amount of carbon emissions. In addition, they demonstrated that the EKC hypothesis is correct. [23] studied the effect of financial development on ecological footprint and investigate the role of institutional quality in the ecological footprint financial development nexus from 1984 to 2017. Employing ARDL models, the findings shows that financial development degrade ecological quality while human capital and institutional quality reduce ecological footprint. Ahmad studied the nexus between economic complexity, institutional quality, economic growth, energy consumption and environmental degradation in emerging countries from 1984 to 2017. Using Cross sectional ARDL model, the findings shows that economic complexity increase environmental degradation while high level of economic complexity mitigate ecological footprint studied the effect of green electricity use, technological innovation, democracy and economic growth on ecological footprint from 1995 to 2018 in six Asian countries. The findings shows that renewable electricity promote ecological quality.

The article "Dose institutional quality influences the relationship between urbanization and CO2 emissions?" was retracted in 2025. Reasons: concerns about the results or conclusions; concerns about the peer review; concerns about the authorship.

### Other factors effecting carbon emission

A vast number of scholars in earlier studies discussed and contested the significance of many aspects in environmental sustainability. These factors have been regarded important in various ways. For instance, [24] explore the relationship between economic growth and technological breakthroughs in the countries of Central and Eastern Europe. They also investigate the relationship between urbanization and the efficiency of governance in these countries. The authors concluded that there is a positive association between innovation and economic growth by using patents, trademarks, and R&D spending as measures of innovation. The effects of technology on the rate of economic growth in 25 developing nations were investigated in [25] study. They found that spending on R&D had a significant negative influence on economic growth in certain of the nations that were included in the study sample. They did this by employing a random coefficient model, as well as R&D and researchers. [26] investigate the correlation between energy and the expansion of the economy. The authors gathered the information from 1993 to 2015 and used the ARDL model in their analysis. According to the findings, economic expansion leads to an increase in the consumption of renewable energy. It was also shown that financial prosperity led to an increase in the utilization of renewable energy. The spatial vector autoregression model was used by [27] to investigate the relationship between economic growth, carbon emissions, and technological innovation from 2003 to 2017. The time period covered by the study was from 2003 to 2017. The findings of this study reveal that there is a positive correlation between the different study factors. [28] also carried out an investigation of this kind utilizing ARDL over the years 1980–2018. The nation of Pakistan served as the focus of the research, and the authors’ findings validated the EKC theory by demonstrating that economic expansion leads to considerable increases in carbon emissions. They provide additional evidence that carbon emissions can be reduced through the use of innovative technology and renewable sources of energy. The rise in carbon dioxide emissions in Pakistan can be attributed in large part to the effects of globalization. The research conducted by [29] investigates the relationship between the consumption of renewable energy, technical innovation, and carbon emissions in Malaysia. The findings imply that adopting renewable energy can assist reduce environmental deterioration, and that technological innovation can lower ecological footprints and carbon emissions. The model used to come to these conclusions was a bootstrapped ARDL model. The EKC theory was validated by their research as well. Using panel-corrected standard errors, generalized least squares, and cointegration methods, [30] investigate the impact of consumption of renewable energy, technological innovation, and information and communications technology (ICT) on carbon emissions in BRICS countries from 1990 to 2019. The authors discovered that two-thirds of the information technology indicators brought about a reduction in emissions, but economic growth and financial development brought about an increase in emissions. The use of renewable energy and technological advancement both had a negative impact on emissions, while rising emissions were determined to be the result of commerce and landline subscriptions. In order to evaluate the innovation Claudia curve and the EKC hypothesis. [31] conducted research on the influence of innovation and consumption of renewable energy sources on carbon emissions in OECD nations. The authors discovered that innovation and economic growth both contribute to a rise in carbon emissions, however foreign direct investment (FDI) has a negative effect on carbon emissions when applied to data from 2004 to 2019. In a similar vein, the influence that renewable energy has on emissions is a negative one; yet, the interactions between innovations and renewable energy continue to have positive benefits. In the same vein, industrialization, energy use, commercialization, and financial development all have a negative impact on the quality of the environment in OECD countries. Using both static and dynamic models, [19] explored the link between foreign direct investment (FDI), energy, and carbon dioxide. The developing world, the global community, and the belt and road initiatives all used the years 2002 to 2019 for their sample data time period. The connection that exists between. The findings indicate that the quality of institutions has a positive impact on foreign direct investment (FDI), although this effect does not hold true for all panels, and high energy usage has a negative impact on FDI inflows. In a similar vein, increased economic expansion is accompanied with a rise in emissions, which provides support for the EKC hypothesis. They discovered varying outcomes in regard to the effect that FDI had on emissions across the various panels. [32] conducted an analysis of the data collected from the belt and road countries from the years 2000 to 2019 using both dynamic and static models. According to the findings, economic expansion, increased reliance on information and communications technology, and increased energy consumption are all factors that are driving up carbon emissions, whereas international trade and the utilization of renewable energy sources are driving down carbon emissions. In a similar vein, several models show that foreign direct investment can either have a positive or negative impact on the amount of carbon dioxide emissions [33] used systematic generalized method of moments models and vector autoregressive models for his research on energy consumption and carbon emissions in Africa. The findings indicated that there was a one-way causative association between coal and mortality, as well as a one-way causal relationship between coal and per capita income and fuel consumption. In a similar vein, a correlation in both directions was discovered between the rate of mortality and the amount of energy used. System GMM models demonstrate that the effects of energy consumption on well-being are complex and multifaceted. For example, increasing use of coal has been shown to decrease unemployment, whilst increased consumption of electricity has been shown to decrease newborn mortality. [34] studied the effect of financial development and trade openness on economic growth in south Asian countries from 1980 to 2017 using panel data models. The findings shows that stock market has a positive effect on economic growth where trade openness, reduce economic growth. Bibi examines the importance of banking sector development to economic growth in four South Asian countries: Sri Lanka, Bangladesh, Pakistan, and India. The Fixed Effect (FE), Difference GMM, and System GMM models were applied to the data set from 1980 to 2017. The study’s findings reveal that a bank-based financial development index composed of private sector credit, board money (M2), and domestic credit given by banks has a significant and favorable effect on economic growth in virtually all scenarios. BiBi Using a global balanced panel data set of 193 upper middle income (UMI), lower middle income (LMI), and high income (HMI) countries from 1998 to 2018, the study for the first time investigates the role of FDI, banks, and stock market financial development on economic growth using static methods and dynamic approaches, contributing to the scarce literature on the collective and across income-based groups of countries. All model findings for the global panel show that FDI has a significant and beneficial effect on economic growth in the global panel, lower medium income (LMI) and upper middle income (UMI) nations, but not in high income (HI) countries. Banking sector development has a considerable but negative impact on economic growth in the global panel, high income and upper middle-income nations, but not in the lower middle-income (LMI) countries. In the worldwide panel, stock market development has a considerable but negative impact on economic growth. [35] discover that monetary policy is in control; the price level has no effect on production or the exchange rate. The only factor that can influence the trend of the exchange rate and the Consumer Price Index is monetary policy. The real policy was a fixed exchange rate, and currency depreciations, such as Japan’s, were extremely successful in terms of stability. The findings suggest that a monetary exchange rate and consumer price index system allows the central bank to stabilize several macroeconomic indices and disruptions. Jamil Using Per Capita GDP, GDP growth, Inflation, and Foreign Trade, the Generalized Method of Movements (GMM) is used to evaluate the impact of exchange rate regimes on economies and macroeconomic stability. The United States Dollar led the world currency by a wide margin. Countries around the world want to see currency impact and exchange rates stabilize. We discover that after Bretton Woods, management shifts from fixed to flexible: There are strong correlations between the choice of exchange rate regime and the growth of countries. [36] studied US recession in 2023 and its economic implications. The authors employed economic models to assess the likelihood of recession. Using Keynesian Cross and IS-LM model, the findings shows the significance of timely and targeted stimulus, the need for coordinated monetary and fiscal policies and the long term structural reform importance. [37] studied the Butterfly effect and its implication for resilience in complex socio ecological systems. This study aims to uncover the nonlinear dynamics, tipping points, and feedback loops that magnify or reduce the consequences of modest perturbations in complex systems by scrutinizing case studies and applying mathematical modelling. Furthermore, it investigates how understanding the Butterfly Effect might influence techniques for increasing the resilience of socio-ecological systems, such as adaptive management, scenario planning, and community participation. The study also investigates the ethical and governance implications of complex systems’ unpredictability and interdependence. It emphasizes the importance of inclusive decision-making procedures that take into consideration varied viewpoints and values. [38] studied the livelihood strategies dimensions for the inhabitants of several occupational groups at Sundarbans, associated cooperatives through sustainable livelihood framework. The study concludes that with the recommendation of Mangrove regeneration at Sundarbans. [39] explore the impact of particulate emission damage, natural resources, growth in agriculture land and population growth on output per worker in Nigeria. Using ARDL model, the findings shows that output per worker increased with an increase in the explained variables used in the study. The findings shows that sustainable growth can be achieved through the reduction of human activities that deplete the environment. [40] examine the manager’s perception about Green Human Resource Management and its practices in the corporate sector of Khyber Pakhtunkhwa (henceforth, KP), Pakistan. The study shows that shows that on average 63 percent of the managers do green practices and 38 percent do not, 64 percent of managers do eco-friendly practices in their industries while 53 percent of managers do not, and 42 percent of managers are working to expand the sphere of green HRM practices but 57 percent of managers do not work as such to expand green HRM practices in their organization. [41] investigated the dynamic effects of financial development, renewable energy utilization, technical innovation, economic growth, and urbanization on carbon dioxide (CO2) emissions in India. Using time series data from 1990 to 2020 using an Autoregressive Distributed Lag (ARDL) model, this study assesses short- and long-run dynamics. The results of the ARDL short- and long-run analyses revealed that financial development, economic expansion, and urbanization have a positive and significant effect on CO2 emissions in India. In contrast, the short- and long-term coefficients for renewable energy utilization and technical innovation are both negative and statistically significant, implying that increasing these variables will result in decreased CO2 emissions. [42] studied the financial availability and innovation link with environmental and firm performance. The results show that suitable financial resources have contributed to the performance of financial instruments, but they also play a significant part in environmental performance. [43] studied the effect of carbon emission, energy use and economic growth on innovations in 181 countries of the world from 1980 to 2019. The findings shows that carbon dioxide and economic growth increase technological innovations while the inflow of FDI decrease innovations output. Energy consumption also negatively affects innovation indicators except for research and development. [44] studied the nexus between energy consumption, forest and industrialization with carbon emission in Russian. Using ARDL model, the findings shows that energy consumption and industrialization raise carbon emission in Russia. [45] conducted a study on Using Laplace series and partial integration in valuing environmental assets and estimating Green GDP. The study concludes with suggestions for future research to further explore the potential of the proposed method and its impact on sustainable development. [46] studied green building practices and energy facility in public libraries in Rivers State. The findings revealed that Rivers state libraries can preserve archives with renewable energy and green building practices, such as solar power, passive ventilation, native landscaping, water-efficient fixtures and regulated humidity. [47] evaluate the potential for adapting the meritocracy, pragmatism, and honesty (MPH) model to the Nigerian context with the aim of promoting economic development in the country. he results of the study suggest that adopting the MPH model in Nigeria could lead to increased economic growth, improved competitiveness, and reduced poverty and inequality. [48] Using the most up-to-date annual data between 1990 and 2019, this study investigated the evidence of the Environmental Kuznets Curve and the Pollution Haven Hypothesis in Bangladesh. The empirical results indicated that the country has an inverted U-shaped Environmental Kuznets Curve and the adverse impact of foreign direct investment on the environment confirmed the validity of the Pollution Haven Hypothesis in Bangladesh. [49] used 260 Pakistan stock exchange-listed firms data from 2011 to 2020 and estimated impact through Regression least square method and GMM. The results of Regression least square and GMM confirmed that the Corporate social environment and environment friendly Co₂ emission have high significant positive impact on Organizational Performance. Social capital role as mediator is highly positive significance that enhances employee’s social, environment Co₂ emission activity and firm outcomes; Indicate corporate social environment, eco-friendly Co₂ emission and social capital have intangible potential Capital of a firm and their significant impact on organizational performance. [50] Dynamic Ordinary Least Squares (DOLS) technique was used to analyze time series data from 1990 to 2021. According to the results of the DOLS estimation, a one-percentage-point increase in economic growth is associated with a 0.24% increase in CO_2_ emissions. Furthermore, increasing the use of renewable energy by 1% is related with a reduction in CO_2_ emissions of 0.81 percent over the long run, as indicated by the coefficient of renewable energy use being negative and statistically significant. [51] investigate the relationship between economic growth, financial development, and energy consumption in South Asian countries for the period 1991–2020. Panel co-integration procedures are used for empirical purposes. However, the long-run results of the Pooled Mean Group reveal that the impact of financial development and economic growth (GDP) on energy consumption is positive and considerable. Based on the Granger causality results of the Vector Error Correction Methodology, the Conservation Hypothesis holds between economic growth (GDP) and energy consumption in the South Asian Region in both the short and long run. Furthermore, the findings suggest that there is a two-way causal relationship between financial development and energy use.

The article "Dose institutional quality influences the relationship between urbanization and CO2 emissions?" was retracted in 2025. Reasons: concerns about the results or conclusions; concerns about the peer review; concerns about the authorship.

## Methodology

### Data and empirical models

This research investigates the relationship between urbanization, institutional quality and carbon dioxide emissions in the Belt and Road initiative countries. The panel data set for the period of 2002 to 2019 was collected form the world development indicator for the Belt and Road Initiative countries detailed in the S1 Appendix, while the world governance indicator is used to collect data for the government effectiveness. In the field of environmental research, numerous studies, like [11] and [30] used this indicator. [52] examined the relationship between institutional quality, economic growth, and foreign direct investment by using panel data to conduct their research. This study uses the methodology proposed [52]for the analysis of panel data, and as a result, the empirical baseline model equation can be stated as follows:

$${ENTQ}_{it}=\beta_{0}+\beta_{1}{URB}_{it}+\beta_{2}{EDU}_{it}+\beta_{3}{INFR}_{it}+\beta_{4}{EG}_{it}+\beta_{5}{IFDI}_{it}+\beta_{6}{INST}_{it}+\beta_{7}{SAG}_{it}+\beta_{8}{LFR}_{it}+{ɛ}_{it}$$ (1)

ENTQ represent the environmental quality where CO2 is used to proxy for environment. CO2 is measured in metric tons per capita. URB is dependent variable used to represent urbanization measured by the proportion of urban population as total pollution. This indicator is used by Chen, Liu [53]. EDU is education while INFR is infrastructure proxy by fixed telephone subscription/100 people. Several studies has used this indicator to proxy for information and communication technology that represent infrastructure [30] however there are some other indicators also been used by this study used fixed telephone subscription to proxy for infrastructure.

GDP is per capita gross domestic product represents economic growth shown by EG and IFDI is the inflow of foreign direct investment. INST represents institutional quality proxy by government effectiveness. There are six institutional quality indicators however this study focus only on government effectiveness as it is closely related to urbanization. SAG is saving while LFR is labor force. The square of urbanization is included to the model to explore the U-shape association between urbanization and carbon dioxide emission. The U-shape nexus allows us to explore that if urbanization increase carbon dioxide emission in the initial stage, and will it negatively affect carbon dioxide emission until its reach a certain level. This is shown in Eq 2 below;

$${ENTQ}_{it}=\beta_{0}+\beta_{1}{URB}_{it}+\beta_{2}{\left(URB\right)}_{it}^{2}+\beta_{3}{EDU}_{it}+\beta_{4}{INFR}_{it}+\beta_{5}{EG}_{it}+\beta_{6}{IFDI}_{it}+\beta_{7}{INST}_{it}+\beta_{8}{SAG}_{it}+\beta_{9}{LFR}_{it}+{ɛ}_{it}$$ (2)

We also believe that there is the moderating role of institutions stated by government effectiveness in the nexus between urbanization and carbon emission, thus it mean that government effectiveness together with urbanization influence carbon dioxide emission. If there is government effectiveness and efficiency will control the harmful effect of urbanization on environmental quality by establishing polices and control over urbanization factors that harm the quality of environment.

The article "Dose institutional quality influences the relationship between urbanization and CO2 emissions?" was retracted in 2025. Reasons: concerns about the results or conclusions; concerns about the peer review; concerns about the authorship.

Its moderating effect is stated by the government effectiveness and urbanization interaction shown as INTR in Eq 3;

$${ENTQ}_{it}=\beta_{0}+\beta_{1}{URB}_{it}+\beta_{2}{\left(URB\right)}_{it}^{2}+\beta_{3}{EDU}_{it}+\beta_{4}{INFR}_{it}+\beta_{5}{EG}_{it}+\beta_{6}{IFDI}_{it}+\beta_{7}{INST}_{it}+\beta_{8}{SAG}_{it}+\beta_{9}{LFR}_{it}+\beta_{10}\left(INTR\right)+{ɛ}_{it}$$ (3)

It is believed that the nexus between the two variables which are urbanization and carbon dioxide is nonlinear and thus a critical value is specific to urbanization, which brings changes to the effect of urbanization on emissions below and above.

Also, there is transformative role of government effectiveness where the urbanization indirectly effect emission though this indicator. Changes in the level of urbanization, the efficiency of the government has been greatly improved. Effective government can help reduce carbon emissions from urbanization. Government activity is seen as a shift in the urbanization channel that affects carbon emissions.

There is a correlation between the rise in urban population and the accompanying rise in carbon dioxide emission [54]. According to [55], urbanization results in a change from rural to urban settings and from an agrarian to an industrial economy. When there is a growth in urbanization, there will also be an increase in the amount of emissions as a result of increased industrialization, production by residents, and improvements in their living conditions. On the other hand, it has been stated that agglomeration in population owing to the rise in urbanization enhances the efficacy of energy consumption and adds to reaching economies of scale. This is because urbanization causes a greater concentration of people [56]. Numerous findings found in the research that came before this one suggest that a higher level of urbanization results in higher levels of carbon dioxide [57]. When discussing the quality of the environment or its deterioration, carbon emissions are typically stated as tons of carbon per person. In a similar vein, it is a widely held belief that the urbanization rate should be treated as an independent variable when analyzing the impact of this factor on carbon emissions.

The article "Dose institutional quality influences the relationship between urbanization and CO2 emissions?" was retracted in 2025. Reasons: concerns about the results or conclusions; concerns about the peer review; concerns about the authorship.

Under the scope of this research project, urbanization was included as an additional indicator of the social welfare of a region. This factor provides an indication of utility: Changes in energy consumption or other resident activities are significantly associated with infrastructure improvements, which may not have a direct influence on CO2 emissions but are strongly associated with those changes. For instance, local governments will be encouraged to take more action to reduce emissions of carbon if there is a greater knowledge of the detrimental impact that carbon emissions have on citizens. In a similar vein, the number of fixed telephone subscriptions that are taken into account per 100 persons demonstrates the rise in economic growth. According to [58] having a solid infrastructure is essential to the successful operation of activities related to foreign direct investment. As a result, it is anticipated that the infrastructure will make a direct contribution to the IED input. owing to the fact that infrastructure not only affects economic activities but also the quality of the surrounding environment.

GDP per person is the standard by which economic expansion is measured [59, 60]. According to earlier research [61] stronger economic growth is associated with an increase in carbon emission as well as an increase in pollution of the environment. In a similar vein, past research has suggested that a rise in economic growth leads to an increase in carbon emission and a decline in the quality of the environment. According to [62], the amount of money earned per individual is a significant factor that determines the amount of carbon dioxide released into the atmosphere. According to the environmental Kuznets Curve, there is a surge in carbon dioxide emissions during the early stages of economic development; but, once a nation reaches a particular level of development, the emission level begins to decrease. This study adds the quadratic function of economic growth to the previous studies in order to examine the non-linear influence of per capita growth on carbon dioxide emission. The previous studies provided the foundation for this investigation. A significant number of studies have considered how foreign direct investment (FDI) affects carbon dioxide levels. This effect can either have a detrimental or beneficial impact, depending on the amount of foreign direct investment (FDI) that comes into a country. The pollution halo theory and the pollution haven effect are the primary vehicles via which the direct investment effect of foreign direct investment is communicated to the public. The pollution haven hypothesis assumes that greater FDI will raise carbon dioxide emissions and deteriorate environmental quality, whereas the halo hypothesis assumes that FDI will reduce carbon emissions and improve environmental quality. According to the first point of view, energy-intensive businesses are more likely to establish their operations in nations that have lax environmental legislation and policies [63]. On the other hand, more recent points of view imply that foreign direct investment (FDI) brings advanced environmental technology and management, hence enhancing environmental quality [64]. We included foreign direct investment in the model to investigate how it would affect the amount of carbon dioxide released.

The article "Dose institutional quality influences the relationship between urbanization and CO2 emissions?" was retracted in 2025. Reasons: concerns about the results or conclusions; concerns about the peer review; concerns about the authorship.

The caliber of the nation’s civil workers, as well as the degree to which political pressure and the autonomy of the bureaucracy, all have a role in determining the extent to which a government is effective. It is another reflection of the dependability of the guarantees provided by the government policies and the quality of the services provided by the government. It overturns the already flexible control that public authorities have even further. The caliber of those who work for the government, the process by which policies are developed, and the manner in which they are carried out all contribute to the efficacy of the government. According to [65] argument, a nation that possesses a plentiful supply of resources has the potential to take use of that supply and, provided that the institutions of the nation operate efficiently, to experience brisk economic expansion. For an economy to experience growth that is both sustainable and consistent over time, it is essential to have governance and institutions that are robust. [66] highlights a variety of government policies that can directly and indirectly affect national economic levels through their impact on market imperfections. These policies can have an effect on economic levels both locally and nationally.

It is possible to view it as a choice between exploiting today and exploiting tomorrow, since it is a means to accumulate money over a period of time and enhance the lives of a number of people in the future. According to the findings of [67] long-term consumer savings are significantly beneficial for the expansion of the economy. In a similar vein, labor is accounted for in the survey due to the impact it has on the quality of the environment. The tables labeled “Tables 1–3” display, in that order, a description of the variables, descriptive statistics, and a correlation matrix for the data, respectively.

The article "Dose institutional quality influences the relationship between urbanization and CO2 emissions?" was retracted in 2025. Reasons: concerns about the results or conclusions; concerns about the peer review; concerns about the authorship.

**Table 1:** Variables description.

Variables description	Symbols
carbon dioxide emissions (metric tons per capita)	CO2
Urbanization has taken as total population	URB
Education attainment compulsory	EDU
Fixed telephone subscription per 100 people	INFR
GDP (Per capita)	EG/GDP
FDI inflow %GDP	IFDI
Government effectiveness (estimate)	INST
Net saving	SAG
Labor force	LFR

**Table 2:** Descriptive statistics.

Variable	Mean	Std. Dev.	Min	Max
CO2	4.481	3.421	0.001	15.047
URB	55.253	16.887	18.19	92.501
EDU	74.901	27.153	0.941	99.882
INFR	19.389	12.376	0.370	51.39
EG	3.984	3.818	-14.75	17.03
IFDI	4.418	6.396	-40.081	60.06
ISNT	.037	.644	-1.23	1.391
SAV	23.815	9.006	-8.290	57.47
LF	3.520	1.22	235	7.90

**Table 3:** Correlation matrix.

	CO2	URB	EDU	FTS	GDP	FDI	GOV	SAV	LF
CO2	1.000								
URB	0.531	1.000							
EDU	0.331	0.173	1.000						
INFR	0.391	0.418	0.360	1.000					
EG	-0.110	-0.053	-0.077	-0.073	1.000				
IFDI	0.064	0.098	0.156	0.104	0.199	1.000			
INST	0.476	0.571	0.255	0.346	-0.104	-0.097	1.000		
SAV	0.261	0.078	-0.125	-0.049	-0.011	-0.141	0.154	1.000	
LFR	-0.032	-0.134	-0.289	-0.168	0.136	-0.057	-0.131	0.475	1. .000

### Econometric models

This study first implemented checking the data stationarity using panel unit root tests. After performing these preliminary tests, formal analysis has been conducted using dynamic and static estimators. These estimators include OLS, fixed-effects models, two-step differencing, and two-step system GMM. This GMM model is [68] and is considered a recent application of the topic, and most studies have focused on this estimator when dealing with panel data. First, the study uses static models, OLS, and fixed effects to deal with heterogeneity. These static estimators were used to compare our findings with previous studies and to compare the results with dynamic model results. By using a GMM model, it will deal with endogeneity issues related to study variables [69]. The system GMM model handles grouping equation differences s at the horizontal level. The instrument specified in the model is the level difference equations delay values. This is the horizontal equation and first difference mean of the study variables. Monte Carlo simulations by [70] indicates that, the most efficient model can be system GMM. Over identifying restriction tests were replaces as the Sargan test which confirm the study model expectations. The values of sargan tests confirm the instruments validity used in the model analysis. The series adjusted test shows whether the hypothesis is confirmed in the second series of correlations of the residuals. In the regression results, the coefficients are validated and the variable variance problem is controlled. With FDI as the dependent variable, the GMM equation can be written as:

$${ENTQ}_{it}=\beta_{0}+\beta_{1}{ENTQ}_{i,t-1}+\beta_{2}Y_{i,t}+{\beta_{3}X}_{i,t}+\varepsilon_{i,t}$$ (4)

In Eq 3, is intendent variable, explanatory variables are shown by Y, and X represent the control variable, *ENTQ*_*i*,*t*-1_ is the first lag of carbon dioxide emission is used as an explanatory variable to measure the effect of the previous year’s emission on the current carbon emission while ε is the error term. The subscripts in the equation specify (i = 1… N) and (t = 2002… 2019) index country and time respectively.

The article "Dose institutional quality influences the relationship between urbanization and CO2 emissions?" was retracted in 2025. Reasons: concerns about the results or conclusions; concerns about the peer review; concerns about the authorship.

## Results and discussions

### Panel unit root tests

Second generation root unit tests are used to check the data stationarity before going the formal analysis. The second-generation test assumes that each series can be subdivided into free cross-sections. Suggested by [71], ADF-enhanced second-generation test based on mean cross-section and first-order difference of a single series to filter cross-sectional correlations due to a single common factor. The unit of origin in each region or country panel is determined by the consistency of the null hypothesis and is therefore tested against conflicting alternatives that allow for regional variation or nation. The second generation of tests from CIPS and CADF are used to test stationery data. The panel root unit test showed that all variables studied were static at the surface or first difference.

The power and ability of the panel unit root test is higher than other unit root tests used for individual time series because it brings together the evidence from the series along with the evidence from the cross-sectional data. Following are tests of all study variables used in all country models. All variables studied were tested at the first difference level and significant values were obtained. As with the second-generation tests show that the variables studied are stationary at levels or first-order differences. In this study, all test results of the panel unit root test strongly supported that the data series were stationary, thus rejecting the null hypothesis of the p-value given the unit root test. All sample countries and all-variables findings are shown in Table 4.

The article "Dose institutional quality influences the relationship between urbanization and CO2 emissions?" was retracted in 2025. Reasons: concerns about the results or conclusions; concerns about the peer review; concerns about the authorship.

**Table 4:** Panel unit root test results.

Variables	CIPS		CADF	
	I(0)	I(1)	I(0)	I(1)
carbon dioxide	-1.667	-3.575 ***	-0.284	-3.831***
URB	-1.629	-2.402***	-2.547***	-2.110**
EDU	-1.810	-4.202***	-1.675	-2.632***
FTS	-3.473***	-2.883***	-3.240**	-3.735***
GDP	-3.641***	-5.167 ***	-3.064***	-4.299***
FDI	-2.888***	-6.063***	-2.481***	-5.294***
GOV	-2.483***	-3.883***	-2.240**	-2.735***
SAV	-1.542	-3.702***	-1.454	-2.328***
LF	-1.901	-4.202***	-1.675	-2.632***

Note:

**, *** shows significance level at 5 percent and 1 percent respectively

### Model results on the effect of urbanization on carbon dioxide emission

The direct impact that urbanization has on carbon emissions is presented in Table 5, together with the results of additional variables that explain the phenomenon. OLS, FE, differential GMM, and two-step systematic GMM were employed for the analysis; nevertheless, this study is primarily concerned with two-step GMM. The Methodology section goes into detail about these various models. The findings from the emissions demonstrate that all of the models have positive and significant coefficients predicted for urbanization. This is because urbanization raises the concentration of carbon dioxide in the sample and lowers the quality of the environment. To be more exact, the parameters in the GMM model predict that CO2 emissions will increase by 0.003% for every 1% growth in urbanization in nations along the Belt and Road. The findings showed that urbanization in the nations that were studied resulted in higher levels of carbon dioxide and contributes to the destruction of the environment. The findings of our investigation are consistent with those of [72]. In addition, they discovered that urbanization leads to an increase in CO2 emissions in the countries of Europe. In a separate piece of research, [73] discovered that the human population had a causal relationship with higher levels of carbon dioxide emissions. According to the findings of yet another investigation [74] urbanization has a considerable impact on the emissions of carbon dioxide.

**Table 5:** The effect of urbanization on carbon emission.

VARIABLES	OLS	FE	DGMM	SGMM
URB	0.048***	0.140***	0.231***	0.003***
	(0.016)	(0.033)	(0.229)	(0.000)
EDU	0.025**	-0.014***	-0.038***	-0.0001***
	(0.010)	(0.012)	(0.084)	(0.001)
FTS	0.000	0.013	0.019	0.0007
	(0.022)	(0.012)	(0.108)	(0.0007)
GDP	-0.032	0.010***	0.040**	0.032***
	(0.043)	(0.007)	(0.014)	(0.002)
FDI	0.027	0.008*	0.003**	0.001**
	(0.028)	(0.005)	(0.011)	(0.001)
GOV	0.290	0.390**	-1.235*	0.025*
	(0.397)	(0.196)	(1.447)	(0.035)
SAV	0.123***	-0.028**	-0.034*	-0.001*
	(0.036)	(0.011)	(0.062)	(0.003)
LF	-8.860	-1.120	-3.830*	5.661
	(1.280)	(1.780)	(2.120)	(1.060)
*CO2*_*i*,*t*-1_			0.218***	0.960***
			(0.304)	(0.0111)
Constant	-3.436**	-1.548		-0.090
	(1.561)	(1.674)		(0.126)
Observations	163	163	112	160
R-squared	0.468	0.434		
Number of id		29	15	29
AR1			0.04 (0.968)	-2.11(0.035)
AR2			-0.21(0.836)	-0.59 (0.554)
Sargan test			109.72(0.307)	137.87(0.770)

Note: Standard errors in parentheses,

*** p<0.01,

** p<0.05,

* p<0.1

According to the findings, education has a negative influence, which is demonstrated by its coefficients; this indicates that education lowers the amount of carbon dioxide emissions. To be more explicit, the two-step system GMM model demonstrates that there will be a reduction in CO2 emissions of 0.001% if there is an increase of one percentage point in the education level of nations that are a part of the BRI. The findings also show that, in order to improve the quality of the environment, it is important to consider the educational attainment of the countries that were sampled.

The article "Dose institutional quality influences the relationship between urbanization and CO2 emissions?" was retracted in 2025. Reasons: concerns about the results or conclusions; concerns about the peer review; concerns about the authorship.

In a similar vein, the infrastructure coefficient is found to be positive but not significant in all of the estimations, indicating that infrastructure likely has a negligible impact on CO2 emissions in the nations that are part of the Belt and Road.

The coefficient for economic growth is considerable but negative, which suggests that it will lead to an increase in carbon dioxide emissions. The expansion of economic activity in the sample countries has a negative impact on the quality of the environment. To be more explicit, the coefficients in the two-step system GMM model predict that an increase in carbon emission will occur if the economies of the countries that are part of the Belt and Road develop by 1%. This will result in an increase of 0.03 percent. According to the findings, an increase in carbon dioxide levels is the root cause of stronger economic growth, which in turn promotes a deterioration of the environment. In line with the findings of [75, 76] the increase in economic growth leading to an increase in emissions is supported by the findings of additional researchers [77]. The quality of the environment suffers as a result of economic growth. [78] contend that there is an upward pressure on ecological footprint due to the expansion of the economy. [79] found the exact opposite outcome. This influence can be linked to the fact that the economies of the countries that are part of the "Belt and Road" initiative are still in the process of developing and emerging and are completely focused on growth. Other economic activity, such manufacturing and industrialization, as well as international trade, also contribute to the expansion of an economy. Hence, the development in economic activity such as manufacturing and industrialization leads to an increase in the demand for energy, and this in turn leads to an increase in the amount of carbon dioxide released. According to these studies, foreign direct investment (FDI) has a beneficial impact on carbon dioxide levels. As a result, an increase in the flow of FDI degrades the quality of the environment. To be more exact, the coefficients in the two-step system GMM model predict that an increase in CO2 emissions of 0.03 percentage points will occur if foreign direct investment (FDI) to nations along the Belt and Road rises by one percentage point. The findings demonstrate that higher levels of foreign direct investment (FDI) into the nations that were investigated lead to higher levels of carbon dioxide emissions and contribute to the deterioration of the environment. According to the findings of [80] foreign direct investment (FDI) led to an increase in carbon emissions, and the link between FDI and carbon emissions was dramatically altered by innovation. It has been demonstrated by [81, 82]. In a similar vein, the efficacy of government yields varying results across models, which suggests that the impact of the effectiveness of government on carbon emissions can be both positive and negative depending on the model. For instance, the estimated coefficients of fixed effects and system GMM are both positive and significant. This suggests that the effectiveness of government has a positive effect on carbon dioxide levels. Emissions are influenced in the opposite direction, and the coefficient is negative in the difference GMM, which indicates that it reduces CO2 emissions. In other words, it has a negative impact on emissions. In the same vein, the coefficients in the OLS model are positive and insignificant, which indicates that the efficiency of the government has no influence on the amount of carbon emissions.

The article "Dose institutional quality influences the relationship between urbanization and CO2 emissions?" was retracted in 2025. Reasons: concerns about the results or conclusions; concerns about the peer review; concerns about the authorship.

The negative significance of savings indicates that savings lead to a reduction in carbon dioxide emissions and an improvement in the quality of the environment in belt countries. The two-step system GMM model demonstrates that if BRI countries save an additional one percentage point of their GDP, this will result in a decrease of 0.001% of their total carbon dioxide emissions. According to the research, one of the most essential things that the countries of the BRI can do to help cut emissions is save money. In a similar vein, the labor coefficient fails to reach statistical significance in the majority of models, which suggests that the effect of labor on carbon emissions is negligible.

### Nonlinear association between urbanization and carbon emission

Table 6 presents the findings of a nonlinear analysis of the association between urbanization and carbon dioxide levels. The calculated coefficient of urbanization is positive and significant, the same as the direct effect model. Urbanization is responsible for a rise in carbon dioxide levels in the countries and highways along the route, as well as a decline in the quality of the environment. To be more exact, the results of the model (system GMM) demonstrate that an increase of one percent in urbanization leads to an increase of 0.018 percent in carbon dioxide. The findings indicate that urbanization in the nations that were studied leads to an increase in carbon dioxide levels and damage of the environment.

**Table 6:** Nonlinear association between urbanization and carbon emission.

VARIABLES	OLS	FE	DGMM	SGMM
**URB**	0.283***	0.106**	13.89**	0.018**
	(0.081)	(0.105)	(5.558)	(0.028)
**URB** ^**2**^	-0.002***	-0.000**	-0.099**	-0.000***
	(0.0007)	(0.001)	(0.041)	(0.000)
**EDU**	0.020**	-0.015**	-0.558**	-0.001**
	(0.009)	(0.012)	(0.239)	(0.001)
	(0.418)	(0.239)	(1.658)	(0.122)
**FTS**	-0.013	0.014	0.192*	0.002*
	(0.022)	(0.012)	(0.099)	(0.003)
**GDP**	-0.027	0.010**	0.0494*	0.048***
	(0.042)	(0.007)	(0.027)	(0.011)
**FDI**	0.032	0.008	0.062*	0.010*
	(0.027)	(0.005)	(0.066)	(0.011)
**GOV**	-0.073**	0.388*	9.564*	0.104*
	(0.406)	(0.197)	(4.578)	(0.108)
**SAV**	0.131***	-0.029**	-0.017	0.0004
	(0.036)	(0.012)	(0.088)	(0.006)
**LF**	-1.510	-1.050	1.730	-5.591
	(1.270)	(1.800)	(1.340)	(1.450)
***CO2***_**i,t-1**_			0.521**	0.948***
			(0.343)	(0.021)
**Constant**	-9.155***	-0.713**		0.494***
	(2.465)	(2.947)		(0.835)
**Observations**	163	163	112	160
**R-squared**	0.497	0.435		
**Number of id**		29	15	29
**AR1**			-0.86(0.391)	-2.07(0.039)
**AR2**			-0.69(0.488)	-0.69(0.488)
**Sargan test**			109.88(0.235)	136.02(0.732)

Note: Standard errors in parentheses,

*** p<0.01,

** p<0.05,

* p<0.1

Yet, the squared coefficient of urbanization demonstrates that there is a negative impact on carbon dioxide after urbanization reaches a particular level. This is the case when urbanization reaches a certain level. According to the findings, estimates of education are shown to be negative and substantial across all models, which suggests that education has the potential to lower carbon dioxide emissions and improve the quality of the environment in nations that are part of the ring. One Belt One Road. To be more explicit, the two-step GMM model demonstrates that there will be a reduction in CO2 emissions of 0.001% if there is an increase of 1 percentage point in the education level of nations that are a part of the BRI. These findings also show that education in the nations that were sampled is necessary in order to improve environmental conditions in such countries. In a similar vein, the coefficient for infrastructure is positive, indicating that there is a considerable rise in the amount of carbon dioxide emissions produced in nations that are part of the Belt and Road. According to the two-step system GMM model, an increase in infrastructure of one percent in the sample countries would lead to an increase in emissions of 0.002 percent.

The article "Dose institutional quality influences the relationship between urbanization and CO2 emissions?" was retracted in 2025. Reasons: concerns about the results or conclusions; concerns about the peer review; concerns about the authorship.

The findings indicate that the estimated coefficient of per capita GDP utilized for economic growth yields a substantial coefficient with a positive sign, which demonstrates that an increase in economic growth results in an increase in the amount of carbon dioxide released. The findings demonstrate that a one percent rise in economic growth will result in a 0.04 percent increase in carbon dioxide levels in the counties, which will have a negative impact on environmental quality.

Foreign direct investment (FDI) has a positive coefficient, which indicates that it contributes to an increase in carbon dioxide emissions and degrades the environmental quality of the country. The findings demonstrate that higher levels of foreign direct investment (FDI) into the sample nations result in higher levels of carbon dioxide emissions and environmental damage. Our findings are consistent with those of [83]; however they are in opposition to the conclusions reached by [80]. The estimated trade openness coefficient has a positive significance in the difference GMM model, indicating that there is a reduction in carbon emissions. However, the estimated trade openness coefficient has a negative significance in the OLS model. This suggests that a rise in commercial activity is associated with an increase in carbon emissions. The findings are in direct contrast to those found by [18].

In a similar vein, all of the other models, with the exception of OLS, find positive values for the government effectiveness coefficients. This conclusion demonstrates that a beneficial effect on carbon dioxide can be attributed to effective government across models. For instance, the predicted coefficient in the two-step GMM model is positive and statistically significant, which indicates that the government’s effectiveness is high. Carbon dioxide emissions have a favorable impact.

According to the findings, the predicted savings coefficients for the different models range from positive to negative, although the effects of labor are not significant. The more a nation’s savings and the larger its labor force, the greater its capacity to produce goods and the greater its output of carbon dioxide. Chen et al. [53] came to a similar conclusion with their research (2019).

The article "Dose institutional quality influences the relationship between urbanization and CO2 emissions?" was retracted in 2025. Reasons: concerns about the results or conclusions; concerns about the peer review; concerns about the authorship.

### The transformative role of government effectiveness

The findings regarding the moderating influence of government efficacy in relation to the urbanization and carbon dioxide emission nexus are presented in Table 7. According to the findings, urbanization leads to higher levels of carbon dioxide emissions and lowers the quality of the environment in the nations that are part in the "Belt and Road" initiative. To be more exact, the coefficients in the two-step system GMM model show that if the rate of urbanization increases by one percent, there will be a 0.001 percent increase in the amount of emissions. According to the findings, urbanization in the nations that were studied led to an increase in carbon dioxide levels and caused environmental deterioration.

**Table 7:** Transformative effect of institutions in the relationship between urbanization and carbon emission.

VARIABLES	OLS	FE	DGMM	SGMM
**URB**	0.178**	0.099**	-3.956	0.001**
	(0.089)	(0.106)	(7.921)	(0.004)
**URB** ^**2**^	-0.001*	0.0003	0.042	-1.650*
	(0.000)	(0.001)	(0.066)	(4.900)
**EDU**	0.024**	-0.016**	-0.210**	-0.001**
	(0.009)	(0.012)	(0.253)	(0.001)
	(0.468)	(0.240)	(5.604)	(0.072)
**FTS**	-0.032	0.016	-0.033*	-0.002**
	(0.023)	(0.013)	(0.197)	(0.001)
**GDP**	-0.023	0.009**	0.048***	0.029***
	(0.041)	(0.007)	(0.016)	(0.003)
**FDI**	0.031	0.008	0.016*	0.003*
	(0.027)	(0.005)	(0.017)	(0.001)
**GOV**	4.107**	-0.272	-10.13	0.632***
	(1.663)	(1.177)	(10.54)	(0.179)
GOV*URB	-0.074**	0.011	0.182	-0.011***
	(0.028)	(0.020)	(0.188)	(0.003)
**SAV**	0.104***	-0.029**	-0.074	0.000
	(0.036)	(0.012)	(0.074)	(0.004)
**LF**	-1.200	-8.660	-8.880	2.621
	(1.250)	(1.830)	(6.410)	(9.311)
***CO2***_**i,t-1**_			0.324***	0.950***
			(0.298)	(0.010)
**Constant**	-6.091**	-0.594**		0.001***
	(2.694)	(2.963)		(0.001)
**Observations**	163	163	112	160
**R-squared**	0.518	0.436		
**Number of id**		29	15	29
**AR1**			-0.04(0.966)	-2.11(0.035)
**AR2**			0.64(0.520)	-0.63(0.532)
**Sargan test**			106.63(0.332)	131.40(0.847)

Note: Standard errors in parentheses,

*** p<0.01,

** p<0.05,

* p<0.1

When urbanization reaches a particular level, there is a negative influence on carbon dioxide levels because the results for squared urbanization reveal that the estimated coefficient is negative. According to the data, countries along the Belt and Road that prioritize education have lower levels of carbon dioxide emissions and higher overall environmental quality. To be more explicit, the two-step system GMM model demonstrates that there will be a reduction in CO2 emissions of 0.001% if there is an increase of one percentage point in the education level of nations that are a part of the BRI. The findings also show that, in order to improve the quality of the environment, it is important to consider the educational attainment of the countries that were sampled.

The article "Dose institutional quality influences the relationship between urbanization and CO2 emissions?" was retracted in 2025. Reasons: concerns about the results or conclusions; concerns about the peer review; concerns about the authorship.

There has been positive economic growth, which indicates that there has been an increase in the amount of carbon dioxide emissions and a decrease in the quality of the environment in nations along the Belt and Road. To be more exact, the coefficients in the GMM model of the two-stage system estimate that a 1% economic growth in nations along the Belt and Road will raise carbon emissions by 0.02%. This is based on the assumption that there will be no other significant changes in the system. According to the findings, an increase in carbon emissions is the root cause of increasing economic expansion, which in turn promotes deterioration of the natural environment. Similar to the findings of [84]. The results confirm that increased economic growth is a driver of increased carbon emissions and a reduction in environmental quality.

Because the countries along the Belt and Road are developing and emerging countries, their economies are still developing in order to improve living standards, reduce poverty, or reduce income inequality. This has a positive impact on carbon emissions, which can be attributed to the fact that these countries are still developing their economies. Industrialization, on the other hand, is associated with an increase in energy demand, which in turn is associated with an acceleration of economic growth. As a result, industrialization is associated with an increase in energy consumption, which in turn accelerates economic growth and has a negative impact on environmental quality.

The findings indicate that the predicted FDI coefficient is positive, and as a consequence, it contributes to an increase in carbon dioxide emissions and a decline in the quality of the environment in the nations that are located along the Belt and Road. The findings showed that higher levels of foreign direct investment (FDI) into the sample countries result in higher levels of carbon dioxide emissions and damage of the environment. Our results are similar to research in [85]. [86] discovered that foreign direct investment (FDI) improves the condition of the environment in Asian countries. According to research done by [87] foreign direct investment led to an increase in the productivity of the nations involved and fueled economic growth. It’s possible that this is due to the fact that the sample countries include LDCs and developing countries, both of which are still committed to the idea of fostering economic growth through the expansion of economic activity. One example of this would be attracting large amounts of foreign direct investment at the expense of the environment. Foreign direct investment (FDI) flows into the sample nations are likely to be investments in polluting industries in host countries with significant CO2 emissions. These findings can be referred to as the pollution haven theory since the influx of foreign investment into the host country pollutes and raises carbon emissions, which in turn lowers the quality of the environment.

The article "Dose institutional quality influences the relationship between urbanization and CO2 emissions?" was retracted in 2025. Reasons: concerns about the results or conclusions; concerns about the peer review; concerns about the authorship.

Our findings are consistent with those of [83] who contend that FDI is responsible for high levels of CO2 emissions. However, the findings of [80] opposing.

The coefficients of the interaction term of governance and urbanization are negative and significant in both OLS and GMM models of the two systems, indicating that governance plays a transformative role in the relationship between urbanization and carbon emissions.

Likewise, the saving coefficient is positive, negative, and insignificant in all models, while labor is insignificant in all models.

## Conclusion and policy recommendation

The focus of this investigation focuses mostly on three different goals. The first part of this study examines the direct impact urbanization along with other explanatory and control variables has on CO2 emissions. The second part of this study examines the nonlinear link between urbanization and carbon dioxide, and the third part of this study examines the effectiveness of governments and their role in moderating the relationship between the two. The data of 39 countries along the belt and road are used for the analysis, and OLS, fixed effects, two-step difference GMM, and two-step system GMM models are used. The time span covered is from 2002 to 2019. In the study, second-generation unit root tests were utilized in order to check for the stationarity of the data. The direct effect that urbanization has on carbon emissions is evidence that urbanization has a negative impact on the quality of the environment. While direct foreign investment and economic expansion are both associated favorably with carbon emissions, saving money has the opposite effect and is associated negatively with carbon emissions.

The results of the model that examines the nonlinear influence of urbanization on carbon emissions demonstrate that urbanization leads to an increase in emissions of carbon dioxide and a decline in environmental quality. The urbanization square term produces a significant and negative coefficient. The data indicate that early stages of urbanization are associated with higher carbon emissions and poorer environmental quality, whereas later stages of urbanization are associated with reduced emissions and improved environmental quality. Education is the single most important factor in cutting carbon emissions, whereas infrastructure, economic growth, and foreign direct investment also have a positive influence in this area. The model’s results on the moderating influence of government efficacy on the link between urbanization and carbon emission show that urbanization and carbon emission have a positive correlation, despite the fact that the coefficient of the square term has a negative value. In a similar vein, economic growth, foreign direct investment, and governance all have a positive association with carbon emission, whereas education and infrastructure both have a negative association with carbon emission and work to reduce emissions. The fact that the interaction terms between urbanization and the efficacy of government have a detrimental impact on carbon dioxide levels demonstrates that governance plays a transformative role in the nexus between urbanization and carbon emission in the countries that are part of the Belt and Road initiative.

The article "Dose institutional quality influences the relationship between urbanization and CO2 emissions?" was retracted in 2025. Reasons: concerns about the results or conclusions; concerns about the peer review; concerns about the authorship.

However, the urbanization process in these countries is beneficial to boot economic growth, which in turn can raise the living standard of the people. The findings show that the level of urbanization in the countries that are a part of the Belt and Road initiative leads to an increase in carbon dioxide emissions. However, the findings of this study show that urbanization and economic growth increase carbon dioxide emission, thus worsening the quality of the environment. The sample countries are predominantly developing and emerging economies that need to increase economic growth in order to raise the living standard. On the other hand, according to the square term, emissions begin to decrease after a nation reaches a particular stage of development and urbanization begins to take effect. The research indicates that urbanization is important for economic growth, and that once it reaches a particular level, there is a reduction in carbon emissions as a result of urbanization. The sample nations also have inadequate rules surrounding foreign direct investment, which is problematic given that foreign direct investment leads to an increase in emissions, which may be the reason why the host countries have polluting sectors. Yet, the increase in awareness and the amount of contribution to environmental quality that results from the improved education in the sample countries contributes to the overall improvement in environmental quality. Most notably, this study reveals that institutions such as government effectiveness play a crucial role in discouraging the unfavorable effects of harmful elements on environmental quality through enacting policies. Government effectiveness can develop policies for economic activities that are favourable to environmental quality. This helps to regulate the flow of foreign direct investment and prevents polluting investments from being made. In a similar vein, the efficiency of government can help reduce the negative effects that urbanization has on carbon dioxide emissions. The findings therefore show that these countries have significant government efficacy to decrease environmental degradation, while encouraging economic growth and mitigating the harmful effects of urbanization on environmental quality. This study is restricted in the sense that it only looks at the sample countries, methodologies, and variables that were used. Future research may undertake such kind of research on additional samples by integrating other institutional quality elements, as well as innovations, to draw more important policy suggestions, as innovation also boosts the efficiency of many economic factors that reduce pollution.

The article "Dose institutional quality influences the relationship between urbanization and CO2 emissions?" was retracted in 2025. Reasons: concerns about the results or conclusions; concerns about the peer review; concerns about the authorship.

## Supporting information

S1 Appendix List of countries. (DOCX)
